This article has been retracted.

# Effectiveness of Chinese Native Culture Education for Improving Undergraduate Nursing Students' Transcultural Self-Efficacy

**DOI:** 10.1155/2022/5813946

**Published:** 2022-07-22

**Authors:** Rong Wang, GongXiang Duan, YuanYuan Wu, YinHua Su, JianZhi Li, Li Liao, Huilan Xu

**Affiliations:** ^1^XiangYa School of Public Health, Central South University, Changsha, Hunan 410001, China; ^2^School of Nursing, University of South China, Hengyang, Hunan 421001, China; ^3^Wuxi Tongren Rehabilitation Hospital, Wuxi, Jiangsu 214000, China

## Abstract

**Aim:**

The aim of this study is to evaluate the impact of Chinese native culture education based on Chinese native culture on the intercultural competence of undergraduate nursing students.

**Method:**

A quasi-experimental design with pretest and posttest was used. We recruited nursing students from 4 classes of the School of Nursing in our hospital in 2016 as research subjects. Undergraduate nursing students (*n* = 79) who completed one semester of education in indigenous Chinese culture completed a demographic questionnaire and the transcultural self-efficacy tool (TSET). Chinese native culture education is the topics related to nursing, consistent with the culture of Chinese patients under the background of Chinese native culture, including the dietary habits, taboos, religions, values, particularly Chinese medicine, and specific diseases. The control group (*n* = 91) was students who did not participate in Chinese native culture education and completed the instrument during the same time frame.

**Result:**

Students who participated in Chinese native cultural education significantly improved their transcultural self-efficacy in three dimensions: cognition, emotion, and practice. Compared with the control group, the students in the cultural education group had higher change scores in three sizes of transcultural self-efficacy.

**Conclusion:**

When strengthening cultural education for undergraduate nursing students, adding content related to Chinese native culture can improve their transcultural self-efficacy and meet the growing cultural needs of patients.

## 1. Introduction

Halloran [1] proposed that culture affects patients' ideas about health and illness and that health care, treatment/healing practices, and cultural values determine how patients behave. Cultural factors are closely related to human beings' physical and psychological status [2]. Transcultural self-efficacy (TSE) among nursing students is crucial for their future careers. Developed countries have led the way in research on culturally congruent care and have made breakthroughs in cultural education to promote knowledge of cultural practices. For instance, nursing educators in the USA have noted the importance of culturally congruent care and have integrated relevant content into the fundamental nursing courses taught to baccalaureate nursing students (National [3]). American educators have also reported positive outcomes of diverse cultural interventions to cultivate students' cultural competence as future practitioners [4].

China is a country composed of ethnic Han and 55 other ethnic minorities, with a population of 1.3 billion. According to the Sixth National Population Census, Chinese ethnic minorities and migrant people have increased by 7,362,627 (6.92%) and 116,995,327 (81.03%), respectively, compared with the numbers reported in the Fifth National Population Census (National Bureau of Statistics of the People's Republic of China [5]. Many cultural differences exist between the ethnic Han and other ethnic minorities, including their folk customs, language, religious beliefs, food habits, and values. Berry and Sabatierb [6] study supported the view that cultural differences exist in countries with domestic migration and those with international migration. Schim, Doorenhos, Miller, and Benkert [7] reported that culturally congruent care requires adapting to nations and ethnic minorities and changing among individuals in native cultures. Marshall [8] viewed each contact with an individual patient as a cultural encounter. Qian and Shen [9] proposed that patients' native languages, local characteristics, folk customs, food habits, and other culture-specific characteristics profoundly influenced their health and nursing practice.

Nevertheless, a study by Zhang [10] showed that the mean scores of clinical nurses on cognitive self-efficacy, affective self-efficacy, and practical self-efficacy in a tertiary hospital in Shanghai were not concordant with those previously mentioned, as necessary to address different demographic characteristics. In a study using semistructured in-depth interviews of 16 nurses, Li [11] concluded that a deficit of cultural knowledge among clinical nurses led to their cultural incompetence. The Chinese National Health and Family Planning Commission, as cited by Chen [12], reported approximately 70,000 disputes between health-care personnel and patients related to cultural differences (e.g., health and life, respect and blasphemy, and passion and offense). Most of these disputes occurred because clinical nurses could not provide culturally congruent care to patients from different cultural backgrounds. Chen, Su, and Ouyang [13] and Zhang [10] attributed clinical nurses' deficiencies in providing culturally congruent care to a lack of cultural competence education on campus.

The purpose of the current study was to evaluate the effect of Chinese native culture education (cultural competence education) based on Chinese native culture for one academic semester (five months) on undergraduate nursing students' transcultural self-efficacy. The questions addressed in the study were the following: (1) Will undergraduate nursing students who participate in a Chinese native culture education have increased transcultural self-efficacy scores? (2) Will undergraduate nursing students who participate in a Chinese native culture education have higher self-efficacy change scores than those who do not participate in this education? (3) Will statistically significant differences in TSE levels be found between the cultural education group and the control group following the artistic interventions?

## 2. Method

### 2.1. Design

This study used a two-group, pretest-posttest, quasi-experimental design to compare undergraduate nursing students who completed a Chinese native culture education (*n* = 79) with those who did not complete a Chinese native culture education (*n* = 91).

### 2.2. Sample and Process

One hundred seventy undergraduate nursing students of grade 2016 in the 5th semester were eligible to participate in the study. Among the students, those who were selected to participate in Chinese local cultural education were assigned to the cultural education group (*n* = 79). The control group (*n* = 91) included those students who had not participated in local Chinese cultural education. Permission to conduct this study was obtained from the University's Human Research Ethics Committee. The informed consent forms were acquired from all students.

A written agreement of collaboration with the course instructors emphasized consistent procedures for data collection. Students in the cultural education and control groups studied in two different classes and lived in separate dormitories. Course instructors distributed the instruments, including a demographic questionnaire, a cover letter describing the study, and an instruction sheet on the tool. Students were asked to complete the tool independently in 20 minutes. The course instructors avoid the study from distracting each other. Students in the study were asked to complete the device before and immediately after the survey. Meanwhile, the control group met the agent.

### 2.3. Instrument

The transcultural self-efficacy tool (TSET) measured students' self-efficacy. It consists of 3 subscales and 83 items: The cognitive subscale has 25 items things, the affective subscale has 30 items, and the practical subscale has 28 items. Respondents rate items using a 10-point scale ranging from 1 (not confident) to 10 (totally sure). Respondents' ratings of 1-2 for more than 80% of the subscale items indicated a low level of TSE, ratings of 3-8 for more than 80% of the subscale items indicated a medium level of TSE, and ratings of 9-10 for more than 80% of the subscale items demonstrated a high level of TSE. The Chinese version of the TSET (CV-TSET) was translated by Chen [12], and permission to use it was obtained before the study. In a survey of nurses using the CV-TSET, Zhang, Chen, and Wang [10] reported a content validity index of 0.95, Cronbach's *α* of 0.99, and subscale alphas ranging from 0.84 to 0.99; its construct validity had been examined and confirmed previously. In the present study, Cronbach's *α* for the real instrument, cognitive subscale, affective subscale, and practical subscale were 0.95, 0.87, 0.93, and 0.90, respectively.

### 2.4. Data Analysis

Data analyses were conducted using SPSS version 20.0 software. Descriptive statistics summarized the demographic data. Due to the limited sample size, nonparametric statistics and independent test sets were calculated to determine variable relationships. The *χ*2 test was also used to analyze whether there were statistically significant differences in TSE's cognitive, affective, and practical levels between the two groups of students at the post-test stage. A two-tailed *P* value less than 0.05 was considered statistically significant.

## 3. Results

### 3.1. Sample Characteristics

Students ranged in age from 18 to 22 years. Seventy-nine students of the cultural education groups had completed Chinese native culture education.  Table 1 shows that the baseline characteristics of the undergraduate nursing students in the cultural education group and control group were not statistically different *P* > 0.05.

### 3.2. Research Question One

Transcultural self-efficacy scores on three subscales increased significantly from pretest to posttest for undergraduate nursing students who completed a Chinese native culture education in the 5th semester. These indicated that students had more confidence in their cognitive, affective, and practical cultural competency after the Chinese native culture education (Table 2).

### 3.3. Research Question Two

As indicated in Table 3, undergraduate nursing students who participated in the Chinese native culture education for one academic semester had significantly changed scores on each subscale compared with those not participating in the cultural education. These indicated that the Chinese native culture education effectively increased the transcultural self-efficacy of undergraduate nursing students.

### 3.4. Research Question Three

As shown in Table 4, most students in the cultural education group had a medium self-efficacy level on the three subscales at the beginning and the end of the 5th semester. Most of the students in the control group also had a medium self-efficacy level on the three subscales at the beginning and the end of the 5th semester. No statistically significant differences in cognitive (*P* = 0.0.556), affective (*P* = 0.485), or practical levels (*P* = 0.670) were found in the cultural education group following the cultural interventions. Nor were statistically significant differences in cognitive (*P* = 0.728), affective (*P* = 0.608) or practical levels (*P* = 0.638) between the cultural education and control groups found at the posttest stage.

## 4. Discussion

The current findings indicated that undergraduate nursing students completing a Chinese native culture education had significant improvements in their transcultural self-efficacy's cognitive, p, practical, and affective aspects after an academic semester. They had the highest score in the affective subscale and the most significant change in the cognitive part because the contents of the Chinese native culture education they participated in related directly to the culture and health care.

The results further supported the premise proposed in the CCC model that TSE was influenced by formalized education and other learning experiences. In other words, self-efficacy is a dynamic construct that changes over time in response to new experiences and information [14]. Furthermore, Jeffreys and Dogan [15] found that one semester with educational and cultural interventions was the sole predictor of TSE changes among nursing students. Cortis [16] also found that appropriate education and clinical experiences helped enhance nursing students' confidence in dealing with patients of diverse cultural backgrounds.

Affective self-efficacy refers to respondents' confidence ratings in dealing with values, attitudes, and beliefs concerning cultural awareness, acceptance, appreciation, recognition, and advocacy. Students in two groups were most confident in their attitudes (affective domain) at both the pretest and posttest stages, which is consistent with the CCC model's assumption. These pretest results can be explained by China's history of having 56 ethnic groups that have lived harmoniously throughout its long process of development as a country. The students in both groups have been taught to be friendly with members of diverse cultures from a young age. In the posttest stage, the effective self-efficacy scores of the students in the cultural education group increased and were higher than those of the students in the control group. Students in the cultural education group might have received guidance in examining and recognizing their similarities to and differences from others. They might have gradually corrected their misunderstandings and doubts about others' values, attitudes, and beliefs, making it easier to accept others' differences.

Cognitive self-efficacy refers to respondents' ratings of their confidence in knowing how cultural factors affected patients from different backgrounds in health-care settings where nurses practiced. Students in the two groups were more confident in their knowledge (cognitive domain) at both the pretest and posttest stages, which was consistent with the research findings of the studies by Lim, Downie, and Nathan [17] and Sarafis and Malliarou [18], but inconsistent with the CCC model's assumptions. These findings might be explained by both groups' intentional or unintentional exposure in the pretest stage to diverse cultural knowledge in their daily lives and during the study. The self-efficacy scores of the students in the cultural education group at the posttest stage increased. The positive outcomes might have been related to the learning strategies used, for example, videos, pictures, literature from cultural journals, recalling personal experiences with Chinese ethnic minorities, small- and large-group discussions with debriefing and summary assessments, and communicating with individuals from various cultures.

Practical self-efficacy referred to respondents' ratings of their confidence in identifying patients' values and beliefs when interviewing patients from different cultural backgrounds. Students in two groups were least confident in their culturally congruent caring skills (practical domain) at both the pretest and posttest stages, which is like the research results of Lim, Downie, and Nathan [17] and Sarafis and Malliarou [18], but inconsistent with the CCC model. As mentioned earlier, the curriculum of Chinese nursing students in 4-year baccalaureate programs usually includes general introductory courses in the first year, <Fundamentals of Nursing> in the sophomore year, professional practices of nursing and clinical probation in the junior year, and ten months of clinical internship in the senior year. This course sequence might explain the lack of cultural practice experiences that might have contributed to deficiencies in students' practical self-efficacy scores in the pretest stage. Because of plenty of time for direct contact with patients through cultural observation and practice in the junior year, the applicable self-efficacy score of the cultural education group increased in the posttest stage. It was higher than that of the control group.

The third research question examined whether there were statistically significant differences in TSE levels following the cultural interventions. No statistically significant differences (*P* > 0.05) in the three TSE levels were found in the intervention group following the artistic interventions nor in the three TSE levels between the two groups in the posttest stage (*P* > 0.05), which is inconsistent with the hypothesis (c) that statistically significant differences would be found in TSE levels between the intervention and comparison groups following cultural interventions. This might be due to the reduced sample sizes of the intervention and comparison groups when they were divided into three (low, medium, and high) levels. Yet, when we compared the self-efficacy levels of the students in the intervention and comparison groups from pretest to posttest, we found that cultural interventions contributed to positive outcomes in that the percentages of students with low TSE levels in the intervention group showed a more significant decrease (cognitive domain, 5.0%; affective domain, 5.1%; and a practical part, 5.1%) relative to those of the comparison group (cognitive domain, 3.3%; affective domain, 2.2%; and practical domain, 2.2%). We also found that cultural interventions contributed to positive outcomes and that the increased percentages of medium TSE levels of students in the intervention group (cognitive domain, 6.3%; affective domain, 3.8%; and practical part, 3.8%) were higher than those in the comparison group (cognitive domain, 1.1%; affective domain, 1.1%; and practical domain, 1.1%). Jeffreys and Dogan's [19] study supported the view that early cultural interventions benefited students with at-risk self-efficacy (low or high) levels and helped them become culturally competent. Jeffreys and Dogan [15] also proposed that the most significant changes and improvements were more likely to be observed in students with low or high self-efficacy levels initially, who received formalized education and clinical practice interventions afterward. Growth and other life experiences among individuals should also lead to an increased percentage of medium TSE levels in the comparison group [17].

As early as 1998, the Holistic Nursing Association of the USA recommended that holistic nursing should center on patients and apply nurses' theoretical knowledge and professional nursing skills to care for and guide patients in meeting their health needs in multiple (i.e., physical, psychological, spiritual, cultural, social, and environmental) dimensions. Although Chinese nurses have also appealed to their colleagues to provide holistic nursing to patients, the current nursing practice in China mainly focuses on treating diseases without implementing culturally congruent care for patients from different cultural backgrounds. Most Chinese universities have briefly introduced concepts related to culturally congruent care instead of offering transcultural nursing as an independent course; therefore, knowledge and awareness of cultural influences have not been recognized in nursing education. The cultural education based on Chinese native culture was insufficient. This study supported the use of the CCC model as a theoretical framework for educating students about cultural competence. It also found that cultural-artistic interventions based on native Chinese culture positively affected nursing students' TSE and provided basic knowledge for Chinese nursing educators to help students develop cultural competence at the baccalaureate nursing level to lay a foundation for them to meet Chinese patients' diverse cultural needs when they become nursing practitioners in the future. It should address gaps in research on changes in nursing students' TSE following artistic interventions based on Chinese native culture. The educators in this study set out to use active learning strategies, including integrating related concepts and ideas about culturally congruent care into lecture content [4], cultural case studies [20, 21], cultural sharing [22], and artistic practice. All these efficient methods were used to promote students' cultural competence, ensuring that basic cultural care concepts were instilled, cultural understanding was achieved, and opportunities to develop cultural care skills were offered.

## 5. Limitations

The current study reported that the cultural interventions positively affected the TSE of undergraduate nursing students. Further research should examine whether artistic interventions affect students' cultural competence. In addition, more research should combine quantitative with qualitative methods (e.g., individual interviews) to evaluate the cultural competence of undergraduate nursing students in a more comprehensive manner.

## 6. Conclusion

This study found that educational interventions based on native Chinese culture helped enhance the cultural competence of undergraduate nursing students. The results supported the notion that students' TSE could be improved through formalized education and culturally relevant learning experiences. However, this study did not find statistically significant differences in TSE levels following cultural interventions. The sample sizes of the intervention and comparison groups, which were reduced by dividing them into three (low, medium, and high) levels, might have interfered with the ability to detect statistically significant differences between them.

## 7. Implications

Nursing educators are in a unique position uniquely positioned to promote the development of cultural competence in undergraduate nursing students. Implementing innovative and evidence-based education is a challenge that can contribute to positive learning outcomes. Although it is urgent to make students competent in culture, ongoing research to understand the teaching-learning process of cultural competency is needed [15]. Undergraduate nursing students are the mainstay of nursing careers in the future. Given the variation of demographic characteristics in China and the coexistence of diverse cultures, Chinese nursing educators must encourage Chinese nursing educators and must promote their exposure to active cultural education in the preregistration stage to ensure better health outcomes for patients.

## Figures and Tables

**Table 1:** Status of sample characteristics.

Items		Cultural education group *n* (%)	Control group *n* (%)	*t*/*χ*2	*P*
Age ($\bar{x}\pm s$)		20.25 ± 0.68	20.235 ± 0.70	1.698	0.091
Gender	Male	2 (2.5%)	5 (5.5%)	0.940	0.332
	Female	77 (97.5%)	86 (94.5%)		
Ethnic group	Han	75 (95%)	85 (93.4%)	0.179	0.672
	Minor	4 (5%)	6 (6.6%)		
Birthplace	Urban	34 (43%)	33 (36.3%)	0.813	0.367
	Rural	45 (57%)	58 (63.7%)		
Religious belief	No	76 (96.2%)	89 (97.8%)	0.379	0.538
	Yes	3 (3.8%)	2 (2.2%)		

Independent test sets were calculated to determine variable relationships.

**Table 2:** Transcultural self-efficacy scores of pretest and posttest for two groups^a^.

Subscale	Group	Pretest		Posttest		*t*	*P*
		Mean	SD	Mean	SD		
Cognitive	Cultural education group	148.25	27.50	187.34	26.78	9.051	≤ 0.001
	Control group	149.69	30.75	151.50	26.04	0.429	0.669
Affective	Cultural education group	199.20	30.09	231.00	27.43	6.942	≤ 0.001
	Control group	195.00	32.70	199.83	30.52	1.030	0.304
Practical	Cultural education group	164.08	32.20	186.96	30.84	4.561	≤ 0.001
	Control group	164.92	33.32	167.16	32.76	0.457	0.648

^a^Cultural education group (*n* = 79) and control group (*n* = 91).

**Table 3:** Comparison of change in TSE Scores from pretest to posttest^a^.

Subscale	Group	Mean	SD	*t*	*P*
Cognitive	Control group	1.98	30.15	8.111	≤0.001
	Cultural education group	38.18	27.67		
Affective	Control group	5.74	29.92	6.485	≤0.001
	Cultural education group	35.45	29.64		
Practical	Control group	2.83	33.41	3.007	≤0.001
	Cultural education group	15.97	21.25		

^a^Cultural education group (*n* = 79) and control group (*n* = 91).

**Table 4:** Result of transcultural self-efficacy levels^a^.

Subscale	Group	Level	Pretest		Posttest	
			*n* %		*n* %	
Cognitive	Cultural education group	Low	11	13.9	7	8.9
		Medium	62	78.5	67	84.8
		High	6	7.6	5	6.3
	Control group	Low	13	14.3	10	11.0
		Medium	72	79.1	73	80.2
		High	6	6.6	8	8.8

Affective	Cultural education group	Low	8	10.1	4	5.0
		Medium	59	74.7	62	78.5
		High	12	15.2	13	16.5
	Control group	Low	10	11.0	8	8.8
		Medium	66	72.5	67	73.6
		High	15	16.5	16	17.6

Practical	Cultural education group	Low	15	19.0	11	13.9
		Medium	60	75.9	63	79.7
		High	4	5.1	5	6.4
	Control group	Low	19	20.9	17	18.7
		Medium	66	72.5	67	73.6
		High	6	6.6	7	7.7

^a^Cultural education group (*n* = 79) and control group (*n* = 91).

## Data Availability

All data was included in the manuscript.

## References

[1] Halloran L. (2009). Teaching transcultural nursing through literature. *The Journal of Nursing Education*.

[2] Campinha-Bacote J., Munoz C. (2001). A guiding framework for delivering culturally competent services in case management. *The Case Manager*.

[3] Health N., Medical Research Council (2006). *Cultural Competency in Baccalaureate in Health: A Guide for Policy, Partnership, and Participation*.

[4] Long T. B. (2012). Overview of teaching strategies for cultural competence in nursing students. *Journal of Cultural Diversity*.

[5] National Bureau of Statistics of the People's Republic of China (2011). Communique on Main Data of Sixth National Population Census of the Peoples’ Republic of China. http://www.stats.gov.cn/tjsj/tjgb/rkpcgb/qgrkpcgb/201104/t20110428_30327.html.

[6] Berry J. W., Sabatierb C. (2009). Acculturation, discrimination, and adaptation among second-generation immigrant youth in Montreal and Paris. *International Journal of Intercultural Relations*.

[7] Schim S. M., Doorenhos A. Z., Miller J., Benkert R. (2003). Development of a cultural competence assessment instrument. *Journal of Nursing Measurement*.

[8] Marshall J. (2003). International and cross-cultural issues: six critical changes for our professions. *Folia Phoniatrica et Logopaedica*.

[9] Qian J. F., Shen L. J. (2015). Lack of transcultural nursing based on native Chinese culture of intern nursing students and countermeasure analysis. *China Higher Medical Education*.

[10] Zhang Y. M., Chen J., Wang Y. M. (2016). Survey of status quo of self-efficacy of transcultural care among nurses in Shanghai city. *Chinese Nursing Research*.

[11] Li J. (2016). *Study of Structure and Development Model of Transcultural in Teriartertiaryy Hospital*.

[12] Chen Z. (2014). How to recognize and build a harmonious relationship between health personnel and patients effectively. http://theory.people.com.cn/n/2014/0714/c40531-25275285.html.

[13] Chen Y., Su L. X., Ouyang M. Y. (2014). Foreign and domestic research of education on transcultural nursing. *Journal of Medicine of China*.

[14] Jeffreys M. R. (2000). Development and psychometric evaluation of the transcultural self-efficacy tool: a synthesis of findings. *Journal of Transcultural Nursing*.

[15] Jeffreys M. R., Dogan E. (2012). Evaluating the influence of cultural competence education on students' transcultural self-efficacy perceptions. *Journal of Transcultural Nursing*.

[16] Cortis J. D. (2003). Culture, values and racism: application to nursing. *International Nursing Review*.

[17] Lim J., Downie J., Nathan P. (2004). Nursing students’ self-efficacy in providing transcultural care. *Nurse Education Today*.

[18] Sarafis P. A., Malliarou M. M. (2013). Cultural self-efficacy of baccalaureate nursing students in a Greek university. *Iranian Journal of Nursing and Midwifery Research*.

[19] Jeffreys M. R., Dogan E. (2010). Factor analysis of the transcultural self-efficacy tool (TSET). *Journal of Nursing Measurement*.

[20] Easterby L. M., Siebert B., Woodfield C. J. (2012). A transcultural immersion experience: implications for nursing education. *The ABNF Journal*.

[21] Ruddock H. C., Turner D. S. (2007). Developing cultural sensitivity: nursing students’ experiences of a study abroad program. *Journal of Advanced Nursing*.

[22] Sommer S. (2001). Multicultural nursing education. *Journal of Nursing Education*.

